# HDAC-inhibitor (S)-8 disrupts HDAC6-PP1 complex prompting A375 melanoma cell growth arrest and apoptosis

**DOI:** 10.1111/jcmm.12345

**Published:** 2014-11-06

**Authors:** Manjola Balliu, Luca Guandalini, Maria Novella Romanelli, Massimo D'Amico, Francesco Paoletti

**Affiliations:** a Department of Experimental and Clinical Medicine, University of FlorenceFirenze, Italy; b NEUROFARBA - Department of Neurosciences, Psychology, Drug Research and Child Health, Section of Pharmaceutical and Nutracetical Sciences, University of FlorenceFirenze, Italy; c Department of Biomedical Experimental and Clinical Sciences, Section of Experimental Pathology and Oncology, University of FlorenceFirenze, Italy

**Keywords:** HDAC-inhibitor (S)-8, A375 human melanoma cells, growth arrest, differentiation, apoptosis, HDAC6, protein phosphatase 1 (PP1), HDAC6-PP1 complex, AKT, *in vivo* toxicity

## Abstract

Histone deacetylase inhibitors (HDACi) are agents capable of inducing growth arrest and apoptosis in different tumour cell types. Previously, we reported a series of novel HDACi obtained by hybridizing SAHA or oxamflatin with 1,4-benzodiazepines. Some of these hybrids proved effective against haematological and solid cancer cells and, above all, compound (S)-8 has emerged for its activities in various biological systems. Here, we describe the effectiveness of (S)-8 against highly metastatic human A375 melanoma cells by using normal PIG1 melanocytes as control. (S)-8 prompted: acetylation of histones H3/H4 and α-tubulin; G_0_/G_1_ and G_2_/M cell cycle arrest by rising p21 and hypophos-phorylated RB levels; apoptosis involving the cleavage of PARP and caspase 9, BAD protein augmentation and cytochrome c release; decrease in cell motility, invasiveness and pro-angiogenic potential as shown by results of wound-healing assay, down-regulation of MMP-2 and VEGF-A/VEGF-R2, besides TIMP-1/TIMP-2 up-regulation; and also intracellular accumulation of melanin and neutral lipids. The pan-caspase inhibitor Z-VAD-fmk, but not the antioxidant N-acetyl-cysteine, contrasted these events. Mechanistically, (S)-8 allows the disruption of cytoplasmic HDAC6-protein phosphatase 1 (PP1) complex in A375 cells thus releasing the active PP1 that dephosphorylates AKT and blocks its downstream pro-survival signalling. This view is consistent with results obtained by: inhibiting PP1 with Calyculin A; using PPP1R2-transfected cells with impaired PP1 activity; monitoring drug-induced HDAC6-PP1 complex re-shuffling; and, abrogating HDAC6 expression with specific siRNA. Altogether, (S)-8 proved very effective against melanoma A375 cells, but not normal melanocytes, and safe to normal mice thus offering attractive clinical prospects for treating this aggressive malignancy.

## Introduction

Histone deacetylases (HDACs) and histone acetyl-transferases (HATs) play an opposite and balanced role in chromatin remodelling and epigenetic regulation of gene expression in several diseases. With regard to cancer, HATs are often functionally inactivated or mutated while HDACs are mostly over-expressed [1–4] and become, therefore, the targets for a range of chemically diverse natural and/or synthetic agents - hydroxamates, cyclic peptides, electrophilic ketones, short-chain fatty acids and benzamides - acting as HDAC inhibitors (HDACi) [5–7]. And indeed, these compounds demonstrated to induce: (i) acetylation of histones, thus allowing chromatin relaxation and proper interaction of transcription factors to DNA as well as of non-histone key regulatory proteins [8]; and furthermore (ii) cell growth arrest and apoptosis in different tumour cells through the generation of reactive oxygen species (ROS), the inhibition of angiogenesis and increase in autophagy [5] and, possibly, the activation/inhibition of additional pathways that have not yet been fully clarified.

It is also worth mentioning that, despite possible significant variation in the action mechanism of HDACi depending on the type of neoplastic model and on the compound used, their greater activity towards malignant cells as compared to normal cells has widely been recognized [4,9]. Therefore, several HDACi have been used in the clinic as either monotherapy or in combination with current chemotherapy [5,10]. Vorinostat [11] was the first HDACi approved by the FDA to treat cutaneous T-cell lymphoma [5,12], but also several other structurally diverse chemical agents such as romidepsin, LAQ824 and MS-275 entered clinical trials to cure various kinds of tumours [4–6].

Previously, we reported a series of new HDACi characterized by a 1,4-benzodiazepine ring (BDZ) hybridized with either SAHA or oxamflatin [13] to yield compounds capable of inducing H3/H4 histone acetylation in cell-based-assays; and especially one, termed (S)-2, displayed interesting anticancer properties towards various subtypes of cultured and primary acute myeloid leukaemia cells [14] and prostate adenocarcinoma cells [15]. In the meantime, we kept screening BDZ-hybrids against various cancer models and another compound, namely (S)-8, has recently emerged during a medicinal chemistry study because of its high activity over a panel of cell-based assays [16]. The present work concern the effects of (S)-8 against human metastatic melanoma cell lines derived from highly lethal neoplasms which are often resistant to most treatments [17]. Also, it is worth noting that patients affected by melanomas diagnosed at late stages of development have poor survival rates that are not sufficiently counteracted by current chemotherapy [18] although advanced immunotherapy has appeared somewhat more promising [19]. Results reported herein aim at describing the anti-tumour properties of (S)-8 on A375 metastatic melanoma cells as the primary model (and also on other melanoma cell lines and normal immortalized melanocytes) and understanding its fine mechanism of action to provide additional pharmacological support for therapy of this heterogeneous and life-threatening human cancer.

## Materials and methods

### Compounds and reagents used in the study

The 1,4-benzodiazepine ring (5-phenyl-1,3-dihydro-2-oxo-benzo[e][1,4]-diazepine) was used as the cap of novel hydroxamic-based HDACi [13]. (S) and (R) N1-hydroxy-N8-(1-methyl-2-oxo-5-phenyl-2,3-dihydro-1H-benzo[e][1,4]-diazepin-3-yl)octanediamide [(S)-8] and [(R)-8] were obtained as reported previously [16] where they are labelled with the number 8. The chiral compounds (S)-8 and (R)-8 (Fig. 1) were dissolved in dimethyl sulfoxide (DMSO; Sigma-Aldrich, St Louis, MO, USA) and stored as 0.1 M stock solutions in the dark at room temperature and added directly to the culture media. The amount of DMSO used as the vehicle did not interfere with drug activities. The antioxidant N-Acetyl-Cysteine (NAC, Sigma-Aldrich), the pan-caspase inhibitor Z-VAD-fmk (R&DSystems, Minneapolis, MN, USA), the phosphatase inhibitors Calyculin A and Okadaic acid, and the pan-deacetylase inhibitor trichostatin A (TSA; Santa Cruz Biotechnology, Santa Cruz, CA, USA) were also used. The WST-1 reagent (Roche Diagnostic GmbH, Mannheim, Germany) was employed to assess cell proliferation in culture. All other chemicals were reagent grade.

**Fig. 1:** Compounds used in this article and their HDACi activity. (**A**) Chemical structures of chiral hydroxamic-based compounds (S)-8 and (R)-8. (**B**) HDACi activity of the two enantiomers was comparatively assessed in A375 melanoma cells which were first seeded in 6-well plates (10^5^ cell/well) and allowed to attach overnight. On the next day cultures were added without/with 5 μM (S)-8 or (R)-8 and maintained for 6, 15 and 24 hrs when cells were detached and extracted by sonication. Cell extracts were normalized for protein content and then processed by Western blot; immunostaining of acetylated forms of histones H3 and H4 as well as of α-tubulin and p53 were revealed with specific antibodies; GAPDH was used as the loading control.

### Cell lines and culture conditions

Human melanoma cell lines such as A375 [gift of B. Stecca, Istituto Toscano Tumori (CRL-ITT), Florence, Italy], Hs-294T and MeWo (from prof L Calorini, Department of Biomedical Experimental and Clinical Sciences, Section of Experimental Pathology and Oncology, Florence, Italy) were maintained in DMEM while the immortalized normal human melanocytes PIG1 (kind gift of C. Le Pool, Loyola University Chicago Maywood, IL, USA) were grown in M254 medium added with human melanocyte growth supplement HMGS2 (Life technologies, Carlsbad, CA, USA). All cell lines were propagated in the presence of 10% foetal bovine serum (EuroClone, Life Science Division, Milan, Italy) and 2 mM L-glutamine at 37°C in 5% CO_2_ humidified atmosphere [20].

### Cell extraction, Western blot, and affinity precipitation of HDAC6-PP1 complex

Harvested cells were re-suspended in a lysis buffer, extracted by sonication and samples, once normalized for protein content, were submitted to western blot as reported elsewhere [20]. Membranes were probed with primary antibodies against acetyl-H3, acetyl-H4 and PP2A (Upstate Biotechnology, Millipore, Bilerica, MA, USA); acetylated α-tubulin and α-tubulin (Sigma-Aldrich) GAPDH, PARP, cleaved caspase-9, pAKT, BAD and HDAC6 (Cell Signaling Technology, Danvers, MA, USA); AKT, p21, PP1, pre-caspase 8 and cytochrome c (Santa Cruz Biotechnology); retinoblastoma (RB; BD Pharmingen, Becton, NJ. USA); anti-His (Life technologies). Suitable peroxidase-conjugated IgG preparations (Sigma-Aldrich) were used as secondary antibodies; the ECL procedure was employed for development. For affinity precipitation of HDAC6-PP1 complex, cell extracts from A375 cultures treated without/with 5 μM (S)-8 for 24 hrs were incubated with 25 μl of a microcystin-LR-Sepharose suspension (Millipore) in Eppendorf vials overnight at 4°C on a rotating platform. After a brief centrifugation, Sepharose beads were washed three times with the lysis buffer; then affinity-precipitated proteins were detached with 30 μl of SDS sample buffer and analysed by Western immunoblot for the presence of PP1 and HDAC6.

### Cell cycle analysis and determination of apoptosis

Cell cycle phases were assessed by the propidium iodide (PI)-hypotonic citrate method; apoptosis was measured by the Annexin-V-Fluos/PI test (Roche Molecular Biochemicals, Mannheim, Germany) with the aid of Becton Dickinson FACSCalibur System (Becton-Dickinson, San Jose, CA, USA) [21].

### Quantification of mitochondrial membrane potential

To determine changes in drug-induced transmembrane mitochondrial membrane potential (Δψm), cells have been stained with JC-1 (Invitrogen, Life Technologies) a cationic dye that exhibits potential-dependent accumulation in mitochondria, indicated by a fluorescence emission shift from green (525 ± 10 nm) to red (610 ± 10 nm). A375 cells (0.5 × 10^6^) were treated without/with 2.5 and 5 μM (S)-8 for 24 hrs and then re-suspended in RPMI 1640 containing 15 μg/ml of JC-1 dye for 30 min. at RT in the dark; after that cells were washed and the fluorescence was measured by flow cytometry. Mitochondria depolarization is specifically indicated by a decrease in the red to green fluorescence intensity ratio [22].

### MIB-1 immunostaining

A375 cells were cultured without/with (S)-8 for 48 hrs onto sterile glass coverslips which were then fixed with −20°C methanol, permeabilized with 0.1% Triton X-100, blocked with 3% BSA and incubated overnight at 4°C with MIB-1 antibody (Dako, Glostrup, Denmark) against the nuclear marker Ki-67 that associated with cell growth [23]. The standard avidin–biotin peroxidase complex technique was used for immunostaining. Pictures were taken with a bright field microscope (Nikon Eclipse, mod. 50i) equipped with a digital camera (DS-5M USB2; Nikon Instruments, Florence, Italy).

### Melanin determination

Melanin content of A375 cells was measured according to Nitoda *et al*. [24]. Cells were kept in culture for 24 hrs at 37°C in 5% CO_2_ atmosphere without/with (S)-8. After 48 hrs cells were washed with PBS, harvested by trypsinization and centrifuged for 10 min. at 1.500 × g. Pellets were then dissolved in 1 M NaOH containing 10% DMSO and incubated for 2 hrs at 80°C. Melanin content was measured spectrophotometrically at 475 nm and expressed as relative absorbance unit/10^5^ cells.

### Oil-Red O staining for neutral lipids

To visualize intracellular neutral lipids, A375 cell cultures were washed with PBS, fixed in cold methanol, then stained with Oil-Red-O (ORO) solution (Sigma-Aldrich) and observed under a bright field microscopy [15].

### Clonogenic assay

A375 cells were first pre-treated with (S)-8 as above for one or two d; then were detached, plated onto new dishes at the density of 300 cell/dish and kept without the drug for additional 7 days. Experiments were terminated by washing cultures with ice cold PBS and counting Giemsa-stained colonies after electronically scanning the entire plate.

### Wound-healing assay

Cells were cultured in 6-cm plates until confluence; then monolayers were scratched using a fine sterile tip to wound the substrate. The medium and debris were washed out and replaced with fresh medium containing increasing drug concentrations. Pictures were taken before and 24 hrs after wounding with the aid of a TMS-F phase-contrast microscope and of a Nikon photocamera E 4500 (Nikon Instruments).

### Gel zymography of MMP-2

Matrix metalloproteinase-2 (MMP-2) activity in A375 conditioned media has carried performed as previously described [25]. Gels were stained in 0.5% Coomassie Blue solution for 2 hrs and destained with 5% acetic acid and 10% methanol (v/v) solution until bands of MMP-2 gelatinolytic activity could be visualized and measured by densitometric analysis with Image J Software.

### Quantitative real-time PCR analysis

QRT-PCR was performed with reverse transcripted cDNA of untreated or drug-treated cells by using the Applied Biosystems 7500HT System according to standard protocols. Fold of MMP-2, TIMP-1, TIMP-2, VEGF-A and VEGF-R2 induction were calculated by the changes of each of their Ct values in treated *versus* untreated cells and normalized to the 18S Ct values. Amplification was performed with the default PCR setting: 40 cycles of 95°C for 15 sec. and of 60°C for 60 sec. using a SYBR Green based detection (SYBR Green Master mix; Applied Biosystems) and the following primers: for MMP-2, forward 5′-AGCACCGCGA-CAAGAAGTAT-3′ and reverse 5′-ATTTGTTGCCCAGGAAAA-GTG-3′; TIMP-1, forward 5′-CCAACAGTGTAGGTCTTGGTGAAG-3′ and reverse 5′-TGTGGCT-CCCTGAACA-3′; TIMP-2, forward 5′-AAGAGTTGTTGAAAGTTGACA-AGCA-3′ and reverse 5′-CGGACCGACCGATTGC-3′; VEGF-A, forward 5′-TGATCC-GCATAATCTGCATGG-3′ and reverse 5′-GCTACTGCCATTCCAATCGAGAC-3′; VEGF-R2, forward 5′-TTCTGGACTCTCTCTGCCT-3′ and reverse 5′-TCCGTCTG-GTTGTCATCTGG-3′; 18S, forward 5′-CGGCTACCACATCAAGGAA-3′ and reverse 5′-GCTGGAATTACCGCGGCT-3′.

### Acute toxicity experiments

CD-1 mice (Primm srl, San Raffaele Biomedical Science Park, 20132 Milano, Italy) were grouped in three groups (5 males + 5 females, each) and injected intraperitoneally (i.p.) with either DMSO as the vehicle or increasing amounts of (S)-8 dissolved in DMSO. Each group received a single injection (0.1 ml) containing no drug (Control) or the drug (T1 = 14.5 mg/kg; T2 = 145 mg/kg; corresponding to ∼0.44 and 4.44 mg/mouse, respectively). After the injection animals were observed individually at least once during the first 30 min., periodically during the first 24 hrs, and daily thereafter for a total of 7 days. Mice were weighed at the start (day 0) and the end (day 7) of experiment, when they were killed by rapid (<30 sec.) replacement of air with 100% CO_2_. Full records were maintained for all the measurements and observations. Samples of soft tissues such as liver, kidney and spleen were fixed in 10% (v/v) phosphate-buffered formalin (PBF, pH 7.4) and embedded in paraffin; bones were also fixed in PBF and then decalcified with acidified ethylenedia-minetetra-acetic acid (EDTA) according to standard procedures before paraffin embedding. Consecutive 2.5–5 μm sections of samples were then stained with Haematoxylin/Eosin and examined under a bright field microscope (Nikon Eclipse, mod. 50i) equipped with a digital camera (DS-5M USB2; Nikon Instruments). Compliance statement to Good Practical of Laboratory (from Primm srl, Dosson di Casier, Treviso, Italy). The present study designated CdS REA/09, has been lead in compliance with the Good Practical of Laboratory and the Standard Operating Procedures of the Test Centre of PRIMM srl (Italian Min. of Health authorization no. 172/268/2005).

### siRNA and plasmid transfection

For siRNA transfections: 2 × 10^5^ cells were seeded in 60 mm culture dishes 16 hrs before transfection with 500 pmol of siRNA using 7.5 μl of Lipofectamine RNAiMAX (Life Technologies). HDAC6-siRNA and control non-targeting siRNA (Life Technologies) were used at the same concentrations. Silencing efficiency was monitored by western blotting at 48 hrs after transfection. For plasmide transfections: 2 × 10^5^ cells were seeded in 60 mm dishes 16 hrs before transfection with 2.5 μg of plasmid PPP1R2 pcDNA4/TO/myc-His A (Abgent, San Diego, CA, USA) - coding for the physiological PP1 inhibitor *i.e*. the protein phosphatase inhibitor 2 (I-2) [26] - using 7.5 μl of Lipofectamine LTX (Life Technologies); 24 hrs after transfection cells were incubated without/with 5 μM drug for additional 24 hrs.

### Statistical analysis

Data were analysed by Student's *t*-test. Significance was assessed by anova followed by Newman–Keuls post-tests using Prism version 4.0 (GraphPad Software, San Diego, CA, USA). The difference among values was considered significant at *P* ≤ 0.05.

## Results

### Compounds used in this work and their efficacy as HDACi

The rationale for generating a series of BDZ-hydroxamate hybrids with HDACi activity was previously described [13], and some specific properties of chiral compounds (S)-8 and (R)-8 (Fig. 1A) were reported in a recent medicinal chemistry study [16]. Briefly, the 5-phenyl-1,4-benzodiazepine ring containing a chiral centre in position three was used as the cap and joined with a suberoyl moiety ending with an hydroxamic function like that of SAHA [11]. The BDZ-hydroxamate hybrids (S)-8 and (R)-8 were first assayed for HDACi activity by using metastatic human melanoma A375 cells as the model. Western blot analyses showed that (S)-8 induced acetylation of H3 and H4 histones and of non-histone protein α-tubulin, while (R)-8 was virtually ineffective (Fig. 1B) thus denoting a marked enantioselectivity between the two enantiomers, the eutomer being the (S)-isoform. Notably, none of the two enantiomers prompted acetylation of p53. Given that acetyl-α-tubulin is a specific substrate for the mainly cytoplasmic class IIb enzyme HDAC6 [27], and acetyl-p53 is the key substrate of nuclear class I enzyme HDAC1 [28], it can be assumed that at least in A375 cell-based assays, HDAC6 and not HDAC1was the primary target of (S)-8.

### (S)-8 and (R)-8 effects on growth and cell cycle of A375 cells are enantioselective

Further evidence of enantioselectivity of (S)-8 *versus* (R)-8 was provided by comparing their effects on growth and cell cycle distribution of A375 cells. In cultures treated with 2.5 and 5 μM (S)-8 for three d, cell growth was fully inhibited, while growth rates in (R)-8-treated cultures overlapped those of the control (Fig. 2A); furthermore, the decrease in viability of (S)-8-treated cells along with incubation was accompanied by an increased amount of fragments recalling typical apoptotic bodies. Moreover, cell cycle progression as measured by flow cytometry showed that a 24 hrs treatment with 2.5 μM (S)-8 led to a marked arrest of cells in G_0_/G_1_ (about 65% *versus* 38% of control), while 5 μM-treated cells underwent a clear blockage in G_2_/M (up 47% *versus* 13% of control). It is interesting to note that this effect has often been observed in cancer cell populations treated with high dosages of other hydroxamic-based HDACi [29]. In addition, (S)-8 caused a marked reduction in cells in S-phase (from 49% of control to 22% and 13% with 2.5 and 5 μM drug, respectively). Conversely, cell cycle profiles of control and (R)-8-treated cells nearly overlapped (Fig. 2B). Consistent with this, western immunoblot analyses showed that (S)-8 caused a significant dephosphorylation of RB and an increase in p21, whereas (R)-8 was almost ineffective (Fig. 2C). These findings pointed clearly to (S)-8 as the eutomer and, from here on out only its biological-molecular effects in melanoma cells will be investigated further.

**Fig. 2:** Biological effects of (S)-8 and (R)-8 on A375 cells. (**A**) Growth curves: A375 melanoma cells were seeded in 6-well plates (10^5^ cell/well) and allowed to attach overnight. The day after increasing concentrations (0–2.5–5 μM) of drugs were added and incubated up to 3 days. Viable cells (trypan blue-negative) were counted daily with the aid of a Bürker chamber and reported as results of a typical experiment out of three. (**B**) For cell cycle analysis companion cultures were incubated for 24 hrs without/with 2.5–5 μM (S)-8 or (R)-8, then cells were detached and incubated for 30 min. with a PI solution to assess by flow cytometry the percentage of PI-stained cells in different cycle phases. (**C**) Cells were treated as above and then processed by Western blot and immunostained for ppRB/pRB and p21; α-tubulin was used as the loading controls.

### (S)-8-induced apoptosis in A375 cells develops *via* an intrinsic caspase-dependent process

The ability of (S)-8 to induce apoptosis in A375 cells was demonstrated by the dose- and time-dependent cleavage of poly(ADP-ribose) polymerase (PARP; Fig. 3A). However, to understand how the process did really develop the effects of the antioxidant NAC and the pan-caspase inhibitor Z-VAD-fmk were separately examined in cultures treated without/with 5 μM (S)-8. The addition of 15 mM NAC to the cultures did not prevent the drug-induced PARP cleavage thus ruling out any role of ROS in mediating cell death. Instead, the addition of 30 μM Z-VAD-fmk contrasted efficiently the drug-mediated cleavage of PARP and of caspase 9, to indicate that apoptosis in A375 cells occurs *via* a caspase-dependent pathway (Fig. 3B). Moreover, caspase 9 fragmentation was dose- and time dependent, while the pre-caspase 8 signal remained steady throughout the incubation regardless of the drug (Fig. 3C). Consistently, (S)-8 activated an intrinsic apototic process including also pAKT dephosphorylation and increased levels of BAD protein (Fig. 3D), drug-induced dissipation of mitochondrial transmembrane potential (Fig. 3E) and a dose-dependent release of mitochondrial cytochrome c into the cytosol (Fig. 3F).

**Fig. 3:** (S)-8 induces apoptosis in A375 cells. (**A**) A375 cells were incubated for the indicated time-points with increasing amounts of (S)-8 (0–2.5–5 μM). Cell extracts were subjected to Western blot analysis and immunodetection for PARP and its cleaved fragment; α-tubulin was used as the loading control. (**B**) Cells were pre-incubated for 2 hrs with Z-VAD-fmk (30 μM) or NAC (15 mM) and then maintained without/with 5 μM (S)-8 for additional 24 hrs. Cell extracts were analysed by Western immunoblot for the cleaved fragment of both PARP and caspase 9; α-tubulin was used as the reference protein. (**C**) A375 cells were incubated for the indicated time-points with increasing amounts of (S)-8 (0, 2.5, 5 μM). Whole-cell extracts were subjected to Western immunoblot to determine pre-caspase 8, cleaved caspase 9 fragment, and (**D**) pAKT, AKT and BAD; α-tubulin and GAPDH, respectively, were used as the loading controls. (**E**) Treatment of A375 cells for 24 hrs with (S)-8 led to a dose-dependent mitochondrial transmembrane potential (ΔΨ) dissipation as determined by the decrease in red/green fluorescence JC-1 ratio. Values have been normalized by using the control signal (only DMSO) as an arbitrary value of 100%. Each bar is the mean of three independent experiments. (**F**) Aliquots of cytosolic extracts from either untreated or treated cells were analysed by Western immunoblot to reveal the drug-induced release of mitochondrial cytochrome c; α-tubulin was used as the reference protein.

### (S)-8 activated multiple pathways in melanoma A375 cells

The response of A375 cells to (S)-8 is complex and characterized by the activation of multiple pathways which each deserve their own synthetic explanation. First, cells maintained without/with 5 μM drug for 48 hrs and then submitted to the Annexin-V/PI assay showed that nearly 40% of the treated population underwent apoptosis (Fig. 4A, top). Second, companion cultures that were immunostained with MIB-1 [23] to evaluate the *in vitro* growth fraction showed a marked decrease in nuclear positivity in drug-treated compared to control cell cultures (Fig. 4A, bottom). Third, treated cultures also underwent a drop in the number of attached cells that became thinner and longer than the control cells, and displayed dendritic-like elongations that are typical of the normal melanocytic phenotype (Fig. 4B, top). Fourth, A375 cells treated as above synthesized and stored both neutral lipids (Fig. 4B, bottom) and melanin (Fig. 4C) thus revealing the pro-differentiative activity of (S)-8. And finally, growth arrest of (S)-8-treated A375 cells was not strictly dependent on the steady presence of the drug. This assumption derived from results of clonogenic assays during which cells were initially grown without/with 5 μM drug for 1 or 2 days, then detached and re-plated into new 10-mm dishes (300 cell/dish) kept for an additional week in drug-free media. The number of colonies in the dishes decreased progressively as a function of pre-treatment thus suggesting that (S)-8 was capable of committing cells to growth arrest or senescence (Fig. 4D).

**Fig. 4:** (S)-8 activates multiple pathways in melanoma A375 cells. (**A**, top) A375 cells were seeded in 6-well plates (10^5^ cell/well) and allowed to attach overnight. The next day cultures were added without/with 5 μM (S)-8 for 48 hrs and then detached and incubated with Annexin-V-Fluos in a HEPES buffer containing PI for 15 min.; the number of apoptotic cells were measured by flow cytometry (FACScan equipment). (**A**, bottom) Companion cultures were also immunostained with MIB-1 to determine variations of cell proliferation in treated *versus* untreated cells. (**B**, top) Phase contrast pictures (magnification ×200) of cultures treated as above showed that (S)-8 caused significant changes in cell density and morphology. (**B**, bottom) Microscopic visualization of the effects of (S)-8 on accumulation of neutral lipid droplets in A375 cells after fixation and staining with a solution of Oil-Red-Oil (ORO) (magnification ×200). (**C**) Total melanin content in A375 melanoma cells were assessed spectrophotometrically following 48 hrs treatment with 5 μM (S)-8 (see Materials and Methods) and expressed as absorbance values at 475 nm/10^5^ cells; each column represents the mean ± SD of three separate determinations. (**D**) For clonogenic assay A375 cells were seeded in 6-well plates (10^5^ cell/well) and allowed to attach overnight. The day after cultures were pre-treated without/with 5 μM (S)-8 for 24–48 hrs. After detachment and counting with a Bürker chamber, viable cells (3 × 10^2^) were re-plated into new 100-mm dishes and kept with the drug-free medium for additional 7 days, when monolayers were washed and stained with Giemsa to count the number of colonies.

### (S)-8 reduces motility, invasiveness, migration and pro-angiogenic potential of A375 cells

Results of the wound-healing assay *in vitro* showed that in untreated cultures the wounded area was fully refilled within 24 hrs, while in drug-treated cultures this process was delayed in a dose-dependent manner (Fig. 5A). Indeed, drug-induced inhibition of HDAC6 led to increased levels of acetyl-α-tubulin that is present in stable microtubules but is absent from dynamic cellular structures [30].

**Fig. 5:** (S)-8 decreases motility, invasiveness, migration and angiogenic potential of A375 cells *in vitro*. (**A**) (S)-8 inhibited A375 cell motility. Confluent cultures were ‘wounded’ with the aid of a sterile plastic tip and maintained without/with increasing amounts of drug for 24 hrs. A phase-contrast microscopy was used to take pictures of the monolayers (magnification ×100). (**B**, left) Aliquots of conditioned media from A375 cultures incubated without/with increasing amounts of (S)-8 for 24 hrs in the absence of FCS were submitted to gelatin zymography and then to densitometric analysis to quantify MMP-2 activity that was reported as% of control. (**B**, right, **C** and **D**) MMP-2, TIMP-1, TIMP-2, VEGF-A and VEGF-R2 mRNA levels, from A375 cells treated without/with 2.5–5 μM (S)-8 for 24 hrs were assessed by quantitative real-time PCR (***P ≤ 0.001).

Moreover, MMPs released in culture by A375 cells were also assayed because of their crucial role in tissue degradation and cell spreading during the metastatic process [31–33]. Conditioned medium of untreated/treated cultures was submitted to gelatin zymography and showed that, upon treatment, activity MMP-2 underwent a dose-dependent decrease (Fig. 5B, right) and this was in keeping with the significant reduction in MMP-2 mRNA levels (Fig. 5B, left). In addition, the expression of MMPs tissue inhibitors such as TIMP-1 and TIMP-2 - known to exert anti-metastatic effects by opposing the activity of MMP-2 and other MMPs [34,35] - was strikingly up-regulated after a 24 hrs treatment (Fig. 5C). At the same time, there was a marked drug-induced down-regulation of VEGF-A and its receptor VEGF-R2 (Fig. 5D), indicating a significant decrease in A375 pro-angiogenic potential.

### (S)-8 prompts growth arrest and apoptosis in different melanoma cell lines but not in normal PIG1 melanocytes and it is safe to normal mice *in vivo*

Anticancer properties of (S)-8, in terms of growth arrest and apoptosis as reported for A375 cells were also assessed in two other metastatic melanoma cell lines, namely Hs-294T and MeWo by using normal immortalized PIG1 melanocytes as control. The treatment with 5 μM drug led to a significant decrease in cell viability (Fig. 6A) and a clear increase in PARP cleaved fragment (Fig. 6B) in all the melanoma cell lines, while it was virtually ineffective in normal PIG1 melanocytes.

**Fig. 6:** *In vitro* effects of (S)-8 in different melanoma cell lines *versus* normal human PIG1 melanocytes; and acute toxicity experiments *in vivo*. (**A**) Viability and growth rates were determined in quadruplicate with the aid of the Roche WST-1 proliferation assay according to manufacturer's instructions. Cells from different melanoma established lines (A375, Hs-294T and MeWo) and normal human melanocyte cell line (PIG1) were treated without/with 5 μM (S)-8 for 24 hrs, and then incubated with WST-1 in a phenol red-free medium; absorbance values of media were measured at 450 nm after 3 hrs of incubation. (**B**) Samples of companion cultures were analysed by Western blot and immunostained for the cleaved PARP fragment taken as an apoptotic marker. (**C**) (S)-8 was apparently no toxic to normal CD-1 mice used as the *in vivo* model for acute toxicity experiments. Animals have been injected *i.p*. once with increasing drug amounts dissolved in 0.1 ml DMSO and killed after a week (see Materials and Methods). All the mice displayed an increase in weight and excellent survival rates all through the experiment regardless of the dosage (top panel). Consecutive 2.5–5 μm sections of samples from liver, bone marrow, kidney and spleen were processed as reported before [14], stained with Haematoxylin/Eosin and examined under a bright field microscope (Nikon Eclipse, mod. 50i) equipped with a digital camera (DS-5M USB2; Nikon Instruments). Pictures (magnification: ×200) reported here concern the histology of organs explanted from mice treated with the higher drug dosage, *i.e*. ∼145 mg/kg, corresponding to about 4.4 mg/mouse (bottom panel).

Moreover, acute toxicity experiments *in vivo* were performed by using normal CD-1 mice as the model. Animals were injected *i.p*. with increasing amounts of (S)-8 dissolved in 0.1 ml DMSO and killed a week later (see Materials and Methods). The mice displayed an increase in weight and good survival rates within the time of the experiment regardless of the dosage (Fig. 6C, top panel). Moreover, histology of liver, bone marrow, kidney and spleen specimens from mice receiving either the vehicle or the higher (S)-8 dosage (145 mg/Kg) showed no drug-related tissue alteration such as cell loss, necrotic areas or other signs of acute toxicity as compared to controls (Fig. 6C, bottom panel).

### (S)-8 triggers apoptosis in A375 cells by dissociating the HDAC6-PP1 complex and releasing the active phosphatase

Having established that (S)-8 induced growth arrest and apoptosis by inhibiting the pro-survival AKT pathway, it became important to identify the upstream molecule/s through which these events could be mediated. Mechanistically, AKT dephosphorylation may occur by the deactivation of upstream kinases or activation of downstream phosphatases such as PP1 and PP2A accounting for more than 90% of serine/threonine phosphatase activity in mammalian cells [36]. The roles of the two phosphatases in drug-mediated AKT dephosphorylation in A375 cells was investigated by treating cultures with (S)-8 given alone or in combination with chemical inhibitors of PP1 or PP2A such as Calyculin A (CA) or Okadaic Acid (OA), respectively. CA prompted a drug-independent decrease in PP1 levels as the result, conceivably, of enhanced degradation of the inhibited phosphatase [37], while OA did not alter the PP2A protein profile relative to control. Furthermore, CA caused a marked increase in pAKT levels and abrogated the drug-induced dephosphorylation of AKT. On the other hand, OA was ineffective, and this indicated that PP1 and not PP2A was the phosphatase directly responsible for dephosphorylation of AKT and the blockage of its downstream pro-survival signalling. Moreover, CA, but not OA, (i) abolished the drug-mediated cleavage of both PARP and caspase 9 thus contrasting the apoptotic process; (ii) maintained the hyperphosphorylated status of RB and down-regulated p21 protein, being these two events that favour rather than oppose cancer cell growth and, lastly, (iii) decreased acetylated levels of histones H3/H4 and α-tubulin (Fig. 7A).

**Fig. 7:** The mechanisms of action of (S)-8 in A375 cells. (**A**) Cells were pre-incubated for 2 hrs with either 50 nM Calyculin A (CA) or 25 nM Okadaic Acid (OA) and then maintained without/with 5 μM (S)-8 for additional 24 hrs. Cell extracts were analysed by Western immunoblot for PP1, PP2A, pAKT, AKT, cleaved PARP, cleaved caspase 9, ppRB/pRB, p21, acetyl-α-tubulin, acetyl-H3 and acetyl-H4; GAPDH was used as loading control. (**B**) Cells were pre-incubated for 2 hrs with either 50 nM CA and then maintained without/with either 5 μM (S)-8 or 0.5 μM TSA for additional 24 hrs. Cell extracts were analysed by Western immunoblot for the cleaved PARP fragment by using GAPDH as the reference protein. (**C**) A375-transfected cells with plasmid PPP1R2 pcDNA4/TO/myc-His A were incubated without/with 5 μM (S)-8 for 24 hrs and cell extracts were submitted to Western blot analysis and immunodetection for His, pAKT, cleaved caspase 9 and p21; GAPDH was used as loading control. (**D**) A375 cells were treated without/with 5 μM drug for 24 hrs. Aliquots of cell lysates were incubated with a microcystin-LR-Sepharose suspension for affinity precipitation (AP) of PP1-containing complexes which were then analysed by Western immunoblot for PP1 and HDAC6 content. (**E**) A375 cells were treated without/with 5 μM (S)-8 for 24 hrs or transfected with HDAC6-specific and scrambled siRNA for 48 hrs. Cell lysates were immunoblotted to detect HDAC6, acetyl-α-tubulin and pAKT; GAPDH was used as loading control.

Also, the CA-mediated effects in A375 cells treated without/with either (S)-8 or TSA have been comparatively examined on the same blot and showed that the chemically-induced inhibition of PP1 activity was capable of abrogating pro-apoptotic potential of both hydroxamic HDACis (Fig. 7B).

In addition, PPP1R2 plasmid-transfected cells - where PP1 activity was partly reduced because of the overexpression of its inhibitor I-2 [26] - became more resistant to drug-induced: pAKT dephosphorylation, the cleavage of caspase 9 and increase in p21 (Fig. 7C). Furthermore, the affinity-precipitation of PP1 with microcystin-LR-Sepharose from cell extracts of cultures treated without/with 5 μM (S)-8 for 24 hrs showed that the PP1 signal was comparable regardless of the treatment. Instead, the amount of HDAC6 co-precipitated with PP1 was significantly lower in treated *versus* untreated cells and this might be because of the drug-induced dissociation of cytosolic HDAC6-PP1 complex (Fig. 7D). Finally, the use of siRNA towards HDAC6 was effective in silencing the expression of the deacetylase and, consequently, of its protein signal, and also in dephosphorylating AKT as it occurred in (S)-8-treated cells (Fig. 7E).

## Discussion

The anticancer properties of the new HDACi (S)-8 towards highly metastatic human melanoma A375 cells have been thoroughly described in the previous section. In brief, we reported the multifaceted response of melanoma cells to the drug including cell cycle arrest, differentiation and caspase-dependent-apoptosis that occur at low micromolar dosages and within relatively short times, whereas normal melanocytes are virtually unaffected. Also, (S)-8 is safe to normal mice *in vivo* up to very high dosages as we reported for hydroxamic-based analogue (S)-2 that, instead of undergoing degradation upon *ip* injection, was capable of reaching the tumor masses on the flanks of immuno-suppressed mice xenografted with prostate cancer cells and contrasting tumor growth [15]. Such a low toxic profile and stability of our BDZ-hybrids is particularly important from a translational point of view as the effectiveness of a given HDACi - in terms of concentration needed to exert a valuable therapeutic anticancer activity - must always cope with its potential toxicity to normal tissues.

Mechanistically, (S)-8 acts by dissociating the cytosolic HDAC6-PP1 complex and allowing the release of PP1 that dephosphorylates AKT thus inhibiting its downstream pro-survival pathway. This mechanism of action was partly well described by Brush *et al*. [36] who reported the effect of the TSA on the stability of the cytosolic complexes between some HDACs and PP1, paying special attention to the HDAC6-PP1 complex. Indeed, this complex is the one sensitively targeted by (S)-8 in A375 cells. Furthermore, Chen *et al*. [38] showed that anticancer effects of HDACis in different tumour cell models closely depend on their ability to dissociate cytosolic HDAC-PP1 complexes and permit the free active PP1 to inhibit the AKT downstream signal.

In addition, chemical and biological properties of the three hydroxamic-based HDACis, namely TSA, SAHA and (S)-8, deserve a brief comment. TSA is a very active pan-deacetylase inhibitor causing the disruption of HDAC-PP1 complexes *in vitro* as we described to occur in (S)-8-treated A375 cells. Action mechanisms appear to be the same for both compounds but (S)-8, although less potent, is definitely more attractive than TSA for *in vivo* use. Regarding SAHA and (S)-8, these compounds carry the same suberoyl chain ending with an hydroxamic moiety such as the zinc-chelating group but differ in the cap. SAHA has a small achiral hydrophilic anilido group, while in (S)-8 there is a bulky lipophilic phenyl-1,4-benzodiazepine ring containing a chiral centre in position 3, which is important for activity [14,16]. These structural differences may explain why the two HDACis display distinct pro-apoptotic mechanisms in solid cancer models: SAHA-mediated effects depend mainly on accumulation of ROS and are counteracted by antioxidants [39,40], while effects of (S)-8 rely on activation of caspase cascade and hence are contrasted by pan-caspase inhibitors.

The results reported herein concern the activities of the novel HDACi (S)-8 used alone, and we are well aware that its full anticancer potential in the clinic may derive from combination therapy with either standard or new antineoplastic agents [10,41]. In fact, to overcome the resistance of BRAF(V600E) melanoma A375 cells to MAPK inhibitors, the combined use of MAPK and histone deacetylase inhibitors has recently been proposed [42]. In this context, it could be intriguing to verify whether (S)-8, that targets the HDAC6-PP1 complex and down-regulates the AKT pathway, could also synergize with RAF–MEK inhibitors and enhance their effects in A375 cells.

Overall, our findings have proven the powerful cytostatic, differentiative and pro-apoptotic properties of (S)-8 in highly metastatic human melanoma cells and its safety in normal mice, thus pointing to this drug as an attractive translational tool in support of current therapy for this very aggressive malignancy.

## References

[1] Marks P, Rifkind RA, Richon VM (2001). Histone deacetylases and cancer: causes and therapies. Nat Rev Cancer.

[2] Kouzarides T (1999). Histone acetylases and deacetylases in cell proliferation. Curr Opin Genet Dev.

[3] Monneret C (2005). Histone deacetylase inhibitors. Eur J Med Chem.

[4] Bolden JE, Peart MJ, Johnstone RW (2006). Anticancer activities of histone deacetylase inhibitors. Nat Rev Drug Discov.

[5] Marks PA, Xu WS (2009). Histone deacetylase inhibitors: potential in cancer therapy. J Cell Biochem.

[6] Mai A, Altucci L (2009). Epi-drugs to fight cancer: from chemistry to cancer treatment, the road ahead. Int J Biochem Cell Biol.

[7] Johnstone RW (2002). Histone-deacetylase inhibitors: novel drugs for the treatment of cancer. Nat Rev Drug Discov.

[8] Glozak MA, Sengupta N, Zhang X (2005). Acetylation and deacetylation of non-histone proteins. Gene.

[9] Dokmanovic M, Marks PA (2005). Prospects: histone deacetylase inhibitors. J Cell Biochem.

[10] Bots M, Johnstone RW (2009). Rational combinations using HDAC inhibitors. Clin Cancer Res.

[11] Marks PA, Breslow R (2007). Dimethyl sulfoxide to vorinostat: development of this histone deacetylase inhibitor as an anticancer drug. Nat Biotechnol.

[12] Marquard L, Poulsen CB, Gjerdrum LM (2009). Histone deacetylase 1, 2, 6 and acetylated histone H4 in B- and T-cell lymphomas. Histopathology.

[13] Guandalini L, Cellai C, Laurenzana A (2008). Design, synthesis and preliminary biological evaluation of new hydroxamate histone deacetylase inhibitors as potential antileukemic agents. Bioorg Med Chem Lett.

[14] Cellai C, Balliu M, Laurenzana A (2012). The new low-toxic histone deacetylase inhibitor S-(2) induces apoptosis in various acute myeloid leukemia cells. J Cell Mol Med.

[15] Laurenzana A, Balliu M, Cellai C (2013). Effectiveness of the histone deacetylase inhibitor (S)-2 against LNCaP and PC3 human prostate cancer cells. PLoS ONE.

[16] Guandalini L, Balliu M, Cellai C (2013). Design, synthesis and preliminary evaluation of a series of histone deacetylase inhibitors carrying a benzodiazepine ring. Eur J Med Chem.

[17] Garbe C, Peris K, Hauschild A (2012). Diagnosis and treatment of melanoma. European consensus-based interdisciplinary guideline–Update 2012. Eur J Cancer.

[18] Finn L, Markovic SN, Joseph RW (2012). Therapy for metastatic melanoma: the past, present, and future. BMC Med.

[19] Tanemura A, Kiyohara E, Katayama I (2013). Recent advances and developments in the antitumor effect of the HVJ envelope vector on malignant melanoma: from the bench to clinical application. Cancer Gene Ther.

[20] Laurenzana A, Cellai C, Vannucchi AM (2005). WEB-2086 and WEB-2170 trigger apoptosis in both ATRA-sensitive and -resistant promyelocytic leukemia cells and greatly enhance ATRA differentiation potential. Leukemia.

[21] Cellai C, Laurenzana A, Bianchi E (2009). Mechanistic insight into WEB-2170-induced apoptosis in human acute myelogenous leukemia cells: the crucial role of PTEN. Exp Hematol.

[22] Salvioli S, Ardizzoni A, Franceschi C (1997). JC-1, but not DiOC6(3) or rhodamine 123, is a reliable fluorescent probe to assess delta psi changes in intact cells: implications for studies on mitochondrial functionality during apoptosis. FEBS Lett.

[23] Gerdes J, Schwab U, Lemke H (1983). Production of a mouse monoclonal antibody reactive with a human nuclear antigen associated with cell proliferation. Int J Cancer.

[24] Nitoda T, Fan MD, Kubo I (2007). Anisaldehyde, a melanogenesis potentiator. Z Naturforsch C.

[25] Leber TM, Balkwill FR (1997). Zymography: a single-step staining method for quantitation of proteolytic activity on substrate gels. Anal Biochem.

[26] Shi Y (2009). Serine/threonine phosphatases: mechanism through structure. Cell.

[27] Lee YS, Lim KH, Guo X (2008). The cytoplasmic deacetylase HDAC6 is required for efficient oncogenic tumorigenesis. Cancer Res.

[28] Luo J, Su F, Chen D (2000). Deacetylation of p53 modulates its effect on cell growth and apoptosis. Nature.

[29] Richon VM, Sandhoff TW, Rifkind RA (2000). Histone deacetylase inhibitor selectively induces p21WAF1 expression and gene-associated histone acetylation. Proc Natl Acad Sci USA.

[30] Hubbert C, Guardiola A, Shao R (2002). HDAC6 is a microtubule-associated deacetylase. Nature.

[31] Liotta LA, Tryggvason K, Garbisa S (1980). Metastatic potential correlates with enzymatic degradation of basement membrane collagen. Nature.

[32] Bernhard EJ, Gruber SB, Muschel RJ (1994). Direct evidence linking expression of matrix metalloproteinase 9 (92-kDa gelatinase/collagenase) to the metastatic phenotype in transformed rat embryo cells. Proc Natl Acad Sci USA.

[33] Tsunezuka Y, Kinoh H, Takino T (1996). Expression of membrane-type matrix metalloproteinase 1 (MT1-MMP) in tumor cells enhances pulmonary metastasis in an experimental metastasis assay. Cancer Res.

[34] Naito K, Kanbayashi N, Nakajima S (1994). Inhibition of growth of human tumor cells in nude mice by a metalloproteinase inhibitor. Int J Cancer.

[35] Hua J, Muschel RJ (1996). Inhibition of matrix metalloproteinase 9 expression by a ribozyme blocks metastasis in a rat sarcoma model system. Cancer Res.

[36] Brush MH, Guardiola A, Connor JH (2004). Deacetylase inhibitors disrupt cellular complexes containing protein phosphatases and deacetylases. J Biol Chem.

[37] Favre B, Turowski P, Hemmings BA (1997). Differential inhibition and posttranslational modification of protein phosphatase 1 and 2A in MCF7 cells treated with calyculin-A, okadaic acid, and tautomycin. J Biol Chem.

[38] Chen CS, Weng SC, Tseng PH (2005). Histone acetylation-independent effect of histone deacetylase inhibitors on Akt through the reshuffling of protein phosphatase 1 complexes. J Biol Chem.

[39] Butler LM, Agus DB, Scher HI (2000). Suberoylanilide hydroxamic acid, an inhibitor of histone deacetylase, suppresses the growth of prostate cancer cells *in vitro* and *in vivo*. Cancer Res.

[40] Xu W, Ngo L, Perez G (2006). Intrinsic apoptotic and thioredoxin pathways in human prostate cancer cell response to histone deacetylase inhibitor. Proc Natl Acad Sci USA.

[41] Jones PA, Baylin SB (2007). The epigenomics of cancer. Cell.

[42] Johannessen CM, Johnson LA, Piccioni F (2013). A melanocyte lineage program confers resistance to MAP kinase pathway inhibition. Nature.

